This article has been retracted.

# An ErChen and YinChen Decoction Ameliorates High-Fat-Induced Nonalcoholic Steatohepatitis in Rats by Regulating JNK1 Signaling Pathway

**DOI:** 10.1155/2017/4603701

**Published:** 2017-06-07

**Authors:** Tian-hong Xie, Jun-xiang Li, Tang-you Mao, Yi Guo, Chen Chen, Ya-fei Han, Xiang Tan, Run-hua Chen

**Affiliations:** ^1^Beijing University of Chinese Medicine, No. 11, North Third Ring East Road, Beijing 100029, China; ^2^Gastroenterology Department, Dongfang Hospital, Beijing University of Chinese Medicine, No. 6, 1st Section, Fangxingyuan, Fangzhuang, Beijing 100078, China

## Abstract

ErChen and YinChen decoction (ECYCD) is an effective traditional Chinese medicine and has been widely used in traditional Chinese medicine to treat nonalcoholic steatohepatitis (NASH), with good curative effects. However, the specific mechanisms underlying these effects are unclear. In this study, we determined the efficacy of ECYCD in a high-fat diet-induced NASH rat model, established by 8-week administration of a high-fat diet. ECYCD was administered daily for 4 weeks, after which the rats were euthanized. The results demonstrated that ECYCD ameliorated high-fat diet-induced NASH, as evidenced by decreased liver indexes, reduced hepatic lipid deposition and liver injury, lower serum biochemistry markers (including low-density lipoprotein), and reduced HOMA-IR scores. Moreover, levels of free fatty acids, tumor necrosis factor, and malondialdehyde were decreased, whereas glutathione was increased in the liver. Serum high-density lipoprotein was also increased in the liver, and ECYCD regulated the c-Jun N-terminal kinase 1 (JNK1) signaling pathway by decreasing the levels of JNK1 protein,* JNK1* mRNA, activator protein- (AP-) 1 protein,* AP-1 *mRNA, and phospho-insulin receptor substrate- (IRS-) 1^ser307^ and increasing phopsho-PKB^ser473^ levels. These results suggested that ECYCD could ameliorate high-fat diet-induced NASH in rats through JNK1 signaling. ECYCD may be a safe therapeutic option for the treatment of NASH.

## 1. Introduction

Nonalcoholic fatty liver disease (NAFLD) is characterized by lipid deposition in hepatocytes and is considered the hepatic manifestation of metabolic syndrome [1]. The incidence of NAFLD is high in Western countries and in the Middle East, Far East, Africa, the Caribbean, and Latin America [2]. NAFLD can develop progressively from simple steatosis to nonalcoholic steatohepatitis (NASH), fibrosis, and cirrhosis [3, 4]. In contrast to NAFLD, NASH also involves inflammation, histological changes, and persistent liver injury. NASH can further develop into liver fibrosis and cirrhosis [5, 6]. Therefore, treatment of NASH is the key for preventing the development from NAFLD to fibrosis and cirrhosis.

Although many factors are involved in the development and pathogenesis of NASH, the “two-hit” model is now accepted by the medical community [7, 8]. The core elements of the “two-hit” model are insulin resistance (IR) and oxidative stress. IR leads to excess hepatic lipid accumulation and hepatic steatosis, which sensitizes the liver to the “second hit.” Oxidative stress then leads to inflammation and persistent liver damage [9]. This “two-hit” model has helped us to elucidate the processes contributing to the development and progression of NASH.

c-Jun N-terminal kinase (JNK) is an important mitogen-activated protein kinase (MAPK). The JNK1 signaling pathway has been shown to play a role in NASH. There are three isoforms of JNK: JNK1, JNK2, and JNK3; these proteins are expressed in tissues that are affected by insulin, such as muscle, liver, and adipose tissue. Previous studies have demonstrated that a variety of stimuli, such as free fatty acids (FFAs), can activate JNK1. After JNK1 is activated, phospho-insulin receptor substrate- (IRS-) 1^ser307^ levels increase owing to binding of activated JNK1 to IRS-1 and inhibition of IRS-1 tyrosine phosphorylation. Phospho-PKB^ser473^ downstream of this pathway then decreases further, resulting in attenuation of the insulin signal transduction pathway. This can eventually cause IR, resulting in hepatic steatosis, which can evolve into NASH (the “first hit”) [10–13]. JNK1 activation also leads to activation of the transcription factor activator protein- (AP-) 1 Y170, which increases the release of proinflammatory cytokines and promotes hepatic inflammation [14, 15], that is, the “second hit” of NASH.

According to the etiology and pathogenesis of NASH, patients may use antidiabetic, lipid-lowering, hepatoprotective, and antihypertensive agents as the main treatment options [16]. However, the available drugs to treat NASH are still not sufficiently effective and are associated with major side effects and long-term safety concerns [17]. Thus, there is an urgent need for the development of novel, safe, effective drugs for the treatment of NASH. Previous studies have revealed the therapeutic effects of integrative medicine in treating patients with glucose and lipid metabolism [18–20]. ErChen and YinChen decoction (ECYCD), which combines ErChen decoction and YinChen decoction, is a traditional Chinese medicine. ErChen decoction is described in the Prescriptions of the Bureau of Taiping People's Welfare Pharmacy, and YinChen decoction is described in the Treatise on Febrile Diseases. ErChen decoction and YinChen decoction are used in traditional Chinese medicine to treat NASH. Our previous studies have shown the efficacy of both ErChen decoction and YinChen decoction in NASH. Both of these treatments are thought to regulate glucose and lipid metabolism, reduce lipid deposition, alleviate IR, and suppress inflammation [20, 21]. ErChen decoction can reduce IRS-1^ser307^ and tumor necrosis factor (TNF) levels in rat livers, and YinChen decoction can increase* IRS-1* mRNA levels and decrease* TNF* mRNA levels in the rat liver [22, 23].

Therefore, in this study, we aimed to combine ErChen decoction and YinChen decoction to investigate whether the obtained ECYCD could regulate the JNK1 signaling pathway and to clarify the mechanisms through which ECYCD treatment affects NASH.

## 2. Materials and Methods

### 2.1. Experimental Animals

A total of 60 adult male Sprague-Dawley rats (12 weeks old; weighing 120 ± 20 g) were purchased from the Animal Breeding Center of the Beijing Adams Beifu Company (Beijing, China). The rats were housed at 22 ± 2°C with a relative humidity of 50–60% and a 12 h light/dark cycle. Before starting the experiment, rats were allowed 7 days to adapt to feeding, with free access to food and sterile water. All animal studies were approved by the Animal Ethics Committee of Beijing University of Chinese Medicine and conducted in accordance with the regulations and guidelines for the care and use of experimental animals of Beijing Laboratory Animal Management.

### 2.2. Therapeutic Agents and Reagents

ErChen decoction was described in the Prescriptions of the Bureau of Taiping People's Welfare Pharmacy and contained 15 g Banxia* (Pinellia ternata)*, 15 g Chenpi (orange peel), 9 g Fuling* (Poria cocos)*, and 4.5 g Gancao (licorice). YinChen decoction was described in the Treatise on Febrile Diseases and contained 18 g YinChen (capillary artemisia), 9 g Zhizi (Cape jasmine), and 6 g Dahuang* (Rheum officinale)*. ECYCD granules containing ECYCD ingredients in equal weights were purchased from the Pharmacy Department of Dongfang Hospital, Beijing University of Chinese Medicine (Beijing, China). Rosiglitazone and Polyenylphosphatidylcholine were also purchased from the Pharmacy Department of Dongfang Hospital, Beijing University of Chinese Medicine. Rosiglitazone can improve the sensitivity of target tissues to insulin and reduce IR by activation of peroxisome proliferator activated receptors (PPARs) in tissues. Polyenylphosphatidylcholine can regulate the oxidative balance, inhibit inflammatory factors, alleviate liver injury, and promote the restoration of liver function. The dose used in the animal experiment was calculated according to the clinical equivalent dose for a 60 kg adult.

### 2.3. Establishment of NASH in Model Rats and Experimental Procedures

Rats were randomly divided into the blank (control, *n* = 10) and experimental groups (*n* = 40). The 10 rats in the control group were fed a normal diet, whereas the 40 rats in the experimental group were fed a high-fat diet (a normal diet supplemented with 2% cholesterol and 10% lard, HFD). Consumption of the high-fat diet for 8 weeks was required for the establishment of NASH. After 8 weeks, the experimental group was divided into four groups (*n* = 10 rats/group): the HFD group, the ECYCD group (7.9 g/kg/day, p.o.), the rosiglitazone group (0.6 mg/kg/day, p.o.), and the Polyenylphosphatidylcholine group (71.0 mg/kg/day, p.o.). The rats were treated orally once a day for 4 weeks; rats in the control group were only given DI water. All rats were weighed once a week, and health status, including eating, drinking, behavior, activity, mental state, and hair condition, was observed every day. After the intervention, all rats were euthanized. We collected abdominal aortic blood and separated the serum in order to monitor blood biochemistry. At the maximum margin of the liver, nine small pieces of liver tissue were collected. One fresh section of liver tissue from each rat was used for preparation of frozen sections, and one was used for hematoxylin and eosin (H&E) staining. The other seven fresh sections of liver tissue from each rat were wrapped in aluminum foil, fixed in liquid nitrogen, and preserved. Sections were cleaned with cold physiological saline and used for analysis of proteins and mRNAs from liver tissue homogenates.

### 2.4. Analysis of Body Weight, Liver Weight, and Liver Index

At the end of the experiment, all rats were weighed and then euthanized by an intraperitoneal injection of 10% chloral hydrate after overnight fasting. Livers from all the rats were immediately removed and weighed after rinsing with ice-cold saline. The liver weight index (%) was calculated as the liver weight/body weight × 100%, as previously described [24].

### 2.5. Measurement of Serum Biochemical Parameters

Blood samples from the rats were collected from the abdominal aortic blood and centrifuged at 1000 ×g for 10 min to separate the serum. Alanine aminotransferase (ALT), aspartate aminotransferase (AST), total cholesterol (TC), triglycerides (TG), low-density lipoprotein (LDL), fasting plasma glucose (FPG), and high-density lipoprotein (HDL) levels were tested using an AU480 automatic biochemical analyzer (Japan Olympus Co., Ltd.), as previously described [25]. Fasting insulin (FINS) levels in the serum were detected by radioimmunoassays, as previously described [26]. Calculations were performed to determine the homeostasis model assessment IR (HOMA-IR) index as follows: HOMA-IR = FPG × FINS/22.5.

### 2.6. Histological Examination

After liver samples were collected, one fresh section of liver tissue from each rat was used to prepare frozen sections. Each section was incubated in liquid nitrogen for 4–10 s prior to staining with Oil Red O (Sigma-Aldrich, St. Louis, MO, USA). The mean optical density (MOD) was calculated to quantify the intracellular lipid deposition, using the image analysis software Image Pro-plus 6.0 (Media Cybernetics, USA). One more fresh section of liver tissue from each rat was fixed by immersion in 10% buffered formalin for paraffin wax embedding prior to staining with H&E. The histological examination was performed by a pathologist blinded to the rats' data. The samples were observed using an Olympus CK40 inverted microscope (Olympus, Tokyo, Japan).

### 2.7. Detection of Glutathione (GSH), Malondialdehyde (MDA), Free Fatty Acids (FFAs), and TNF in Liver Tissue

After liver tissues were collected from rats, GSH, MDA, FFA, and TNF levels in the liver tissues were tested using commercially available rat enzyme-linked immunosorbent assay (ELISA) kits (Thermo Fisher Scientific, USA), according to the manufacturer's instructions. Briefly, the samples were diluted to 1 : 10 with normal saline, and the liver tissue was homogenized using an electric homogenizer. Then, the homogenate was centrifuged for 10 min at 45,000 ×g at a temperature of 4°C. The supernatant was extracted to determine the concentration of protein. The absorbance was read at 450 nm using a microplate reader (MULTISKAN MK3, Thermo Fisher Scientific, USA).

### 2.8. Detection of the mRNA Expression Levels of JNK1, AP-1, IRS-1, and PKB by Real-Time Polymerase Chain Reaction (PCR)

Evaluation of mRNA expression was performed using real-time PCR, as previously described [27]. Total RNA was isolated from the liver tissues of the rats using extraction kits (CWbio, Beijing, China). The RNA template was converted to cDNA, using reverse transcription kits (CWbio). After reverse transcription, PCR amplification was performed using SYBR PCR Mixture (CWbio). The primer sequences of target genes were as follows: forward, 5′-TGCTGGTGATAGATGCGTCC-3′, and reverse, 3′-CATTGACAGACGGCGAAGAG-5′, for* JNK1*; forward, 5′-GCCCGGCTAGAGGAAAAAGT-3′, and reverse, 3′-CTGCGTTAGCATGAGTTGGC-5′, for* AP-1*; forward, 5′-AAACCTCCTGTTGAGAGCGG-3′, and reverse, 3′-TGTTGGAATCTCCCACTGGC-5′, for* IRS-1*; forward, 5′-CACCTTCCATGTGGAAACGC-3′, and reverse, 3′-CTCCTGCCGTTTGAGTCCA-5′, for* PKB*. For real-time PCR, the cycling conditions were as follows: 95°C for 10 min, 45 cycles of 95°C for 10 s, and 59°C for 60 s, followed by a melting curve analysis-based assay with conditions of 95°C for 15 s and 72°C for 15 s, with an increase in temperature to 95°C for 15 s. Relative expression was assessed by calculating the expression relative to that of glyceraldehyde 3-phosphate dehydrogenase (GAPDH). The 2^−ΔΔCt^ method was applied for data analysis.

### 2.9. Detection of JNK1, AP-1, IRS-1, Phospho-IRS-1^ser307^, PKB, and Phospho-PKB^ser473^ Levels in the Liver Using Western Blot Analysis

Western blot analysis was conducted as described previously [28]. Proteins were separated from ice-cold liver tissues, and protein concentrations were determined using the bicinchoninic acid assays (Cwbiotech, Beijing, China). Proteins were loaded onto 5–10% gels, separated by sodium dodecyl sulfate polyacrylamide gel electrophoresis (SDS-PAGE), and transferred to polyvinylidene difluoride membranes (Millipore) for 90 min at 300 mA. The membranes were then incubated in blocking buffer for 1.5 h prior to the addition of primary antibodies, including anti-JNK1 (dilution, 1 : 1000), anti-AP-1 (dilution, 1 : 400) antibodies, anti-IRS-1 (dilution, 1 : 500), phospho-IRS-1^ser307^ (dilution, 1 : 1000), anti-PKB (dilution, 1 : 1000), and anti-phospho-PKB^ser473^ (dilution, 1 : 2000). Membranes were incubated at 4°C overnight, washed three times for 10 min, and incubated with secondary antibodies (goat anti-rabbit immunoglobulin G, 111-035-003, and goat anti-mouse immunoglobulin G, 115-035-003 [Jackson Laboratory, USA], and rabbit anti-goat immunoglobulin G, ZB-2306 [ZSGB-BIO, China]). Finally, densitometry was used to quantify protein band intensities using a Gel Image System ver. 4.00 (Tanon, China).

### 2.10. Statistical Analysis

All data are expressed as means ± standard deviations (SDs) and were analyzed by SPSS software version 17.0 (SPSS, Inc., Chicago, IL, USA). Comparisons between the groups were analyzed for statistical significance by one-way analysis of variance and Wilcoxon's signed-rank test. Differences with *P* values of less than 0.05 were considered statistically significant.

## 3. Results

### 3.1. Effects of ECYCD on Body Weight, Liver Weight, and Liver Index in NASH Rats

All animals showed no signs of poor health, and no early deaths occurred. After 8 weeks of the high-fat diet, body weights of the rats consuming the high-fat diet started to increase. By week 12, the weight increase of rats in the HFD group was significantly higher than that in the control group (609.74 ± 51.16 g versus 549.50 ± 36.25 g, resp.; *P* < 0.05). In contrast, significantly reduced weight increases were observed in the ECYCD (551.55 ± 55.41, *P* < 0.05), rosiglitazone (556.10 ± 58.87 g, *P* < 0.05), and polyenylphosphatidylcholine groups (560.28 ± 48.31 g, *P* < 0.05; Figure 1(a)). However, there were no differences among the three groups.

By week 12, the liver weight increase in rats in the HFD group was significantly higher than that in the control group (24.13 ± 4.97 g versus 13.07 ± 1.09 g, resp.; *P* < 0.01). Compared with the HFD group, reduced increases in liver weights were observed in the ECYCD (18.62 ± 3.71 g, *P* < 0.05), rosiglitazone (18.26 ± 4.47 g, *P* < 0.05), and polyenylphosphatidylcholine groups (18.64 ± 4.41 g, *P* < 0.05). However, there were no differences among these three groups (Figure 1(b)).

By week 12, the liver index of rats in HFD group was significantly increased compared with that in the control group (3.96 ± 0.618 versus 2.35 ± 0.099, resp.; *P* < 0.01). Compared with the HFD group, the liver indexes were significantly reduced in the ECYCD (3.34 ± 0.382, *P* < 0.05), rosiglitazone (3.24 ± 0.510, *P* < 0.05), and polyenylphosphatidylcholine groups (3.31 ± 0.525, *P* < 0.05). However, there were no differences among the three groups (Figure 1(c)).

### 3.2. Effects of ECYCD on Histological Changes in the Liver

According to the results of H&E staining, the livers of rats in the control group showed an intact cellular structure (Figure 2(a)). Additionally, compared with the control group, the HFD group showed typical macrovesicular steatosis, ballooned hepatocytes, and inflammatory infiltration with extensive lipid deposition, indicating that the model was successfully established (Figure 2(a)). However, these pathological changes were obviously reduced in the three treatment groups (Figure 2(a)).

Intracellular lipid deposition in hepatocytes was clearly observed by Oil Red O staining (Figure 2(b)). Livers in the HFD group showed significant intracellular lipid deposition compared with those in the control group (0.968 ± 0.139, *P* < 0.01, Figure 2(c)). However, a lesser degree of lipid deposition in hepatocytes was observed in the ECYCD, rosiglitazone, and polyenylphosphatidylcholine groups compared with that in the HFD group (0.150 ± 0.068, 0.172 ± 0.079, and 0.183 ± 0.093, resp.; *P* < 0.01; Figure 2(c)).

### 3.3. Effects of ECYCD on Serum Levels of ALT and AST in NASH Model Rats

Compared with the control group, serum ALT and AST levels in the HFD group increased significantly (ALT: 148.70 ± 45.90 U/L in the HFD group versus 60.90 ± 30.61 U/L in the control group, *P* < 0.01; AST: 463.10 ± 151.08 U/L in the HFD group versus 186.90 ± 36.10 U/L in the control group, *P* < 0.01). ECYCD significantly inhibited the increase in serum levels of ALT and AST compared with the HFD group (ALT: 92.50 ± 43.16 U/L, *P* < 0.05; AST: 255.00 ± 54.95 U/L, *P* < 0.01). Similarly, compared with the HFD group, serum ALT and AST were reduced after treatment with rosiglitazone (ALT: 105.90 ± 33.38 U/L, *P* < 0.05; AST: 314.50 ± 77.31 U/L, *P* < 0.05) and polyenylphosphatidylcholine (ALT: 72.90 ± 25.10 U/L, *P* < 0.01; AST: 224.10 ± 56.08 U/L, *P* < 0.01; Figure 3).

### 3.4. Effects of ECYCD on Serum Levels of TG, TC, HDL, and LDL in NASH Model Rats

Compared with the control group, serum TG, TC, and LDL levels were significantly increased in the HFD group (TG: 1.45 ± 0.235 mM in the HFD group versus 0.535 ± 0.145 mM in the control group, *P* < 0.01; TC: 2.46 ± 0.34 mM in the HFD group versus 1.41 ± 0.21 mM in the control group, *P* < 0.01; LDL: 0.736 ± 0.151 mM in the HFD group versus 0.331 ± 0.052 mM in the control group, *P* < 0.01). Additionally, serum HDL levels were significantly decreased (0.746 ± 0.084 mM in the HFD group versus 1.25 ± 0.130 mM in the control group, *P* < 0.01). Compared with the HFD group, ECYCD caused significant reductions in the increased serum levels of TG, TC, and LDL (TG: 0.592 ± 0.113 mM, *P* < 0.01; TC: 1.72 ± 0.41 mM, *P* < 0.01; LDL: 0.526 ± 0.110 mM, *P* < 0.01). Moreover, serum HDL levels were significantly decreased (HDL: 0.987 ± 0.135 mM versus the HFD group, *P* < 0.01). Significant inhibition of the increases in TG, TC, and LDL and significant inhibition of the decreases in HDL were also observed for rosiglitazone (TG: 0.527 ± 0.113 mM versus the HFD group, *P* < 0.01; TC: 1.66 ± 0.34 mM versus the HFD group, *P* < 0.01; LDL: 0.543 ± 0.102 mM versus the HFD group, *P* < 0.01; HDL: 1.03 ± 0.184 mM versus the HFD group, *P* < 0.01) and polyenylphosphatidylcholine (TG: 0.675 ± 0.175 mM versus the HFD group, *P* < 0.05; TC: 1.96 ± 0.42 mM versus the HFD group, *P* < 0.05; LDL: 0.556 ± 0.105 mM versus the HFD group, *P* < 0.01; HDL: 0.889 ± 0.134 mM versus the HFD group, *P* < 0.05; Figure 4).

### 3.5. Effects of ECYCD on Serum Levels of FPG, FINS, and HOMA-IR in NASH Model Rats

Compared with the control group, the serum levels of FPG and FINS in the HFD group were significantly increased (FPG: 8.42 ± 2.13 mM in the HFD group versus 6.05 ± 1.68 mM in the control group, *P* < 0.05; FINS: 231.91 ± 104.27 *μ*IU/mL in the HFD group versus 109.75 ± 41.42 *μ*IU/mL in the control group, *P* < 0.01). Additionally, HOMA-IR was also increased obviously as compared with that in the control group (76.94 ± 25.37 in the HFD group versus 29.20 ± 12.36 in the control group, *P* < 0.01). With the administration of ECYCD, rosiglitazone, and polyenylphosphatidylcholine, the serum levels of FPG (6.25 ± 1.57, 6.24 ± 1.05, and 6.54 ± 1.41 mM, resp., versus the HFD group, *P* < 0.05, *P* < 0.05, and *P* < 0.05, resp.) and FINS (132.72 ± 34.98, 117.80 ± 26.35, and 143.39 ± 31.25 *μ*IU/mL, resp., versus the HFD group, *P* < 0.05, *P* < 0.01, and *P* < 0.05, resp.) decreased significantly compared with those in the HFD group. Additionally, HOMA-IR (38.90 ± 20.16, 33.57 ± 12.78, and 42.03 ± 13.91, resp., versus the HFD group, *P* < 0.01, *P* < 0.01, and *P* < 0.01, resp.) also decreased significantly compared with that in the HFD group (Figure 5).

### 3.6. Effects of ECYCD on the Levels of GSH, MDA, FFAs, and TNF in Liver Tissue

In the HFD group, the levels of MDA, FFAs, and TNF in the liver increased significantly as compared with those in the control group (MDA: 13.23 ± 2.61 ng/mL in the HFD group versus 7.24 ± 2.34 ng/mL in the control group, *P* < 0.01; FFAs: 1.791 ± 0.487 *μ*g/mL in the HFD group versus 0.560 ± 0.373 *μ*g/mL in the control group, *P* < 0.01; TNF: 218.64 ± 31.36 pg/mL in the HFD group versus 93.63 ± 56.40 pg/mL in the control group, *P* < 0.01). GSH levels in the livers of the HFD group decreased significantly as compared with those in the control group (GSH: 4.17 ± 1.30 ng/mL in the HFD group versus 9.71 ± 2.62 ng/mL in the control group, *P* < 0.01).

After oral administration of ECYCD, rosiglitazone, and polyenylphosphatidylcholine for 4 weeks, the levels of MDA, FFAs, and TNF in the livers decreased significantly compared with those in the HFD group (MDA: 9.27 ± 2.39, 10.39 ± 2.12, and 8.32 ± 1.48 ng/mL, resp., versus the HFD group *P* < 0.01, *P* < 0.05, and *P* < 0.01, resp.; FFAs: 1.139 ± 0.56, 0.864 ± 0.343, and 1.06 ± 0.558 *μ*g/mL, resp., versus the HFD group *P* < 0.05, *P* < 0.01, and *P* < 0.01, resp.; TNF: 141.29 ± 59.74, 166.09 ± 51.34, and 131.82 ± 42.05 pg/mL, resp., versus the HFD group *P* < 0.01, *P* < 0.05, and *P* < 0.01, resp.). Additionally, GSH levels were increased in the livers of these rats (6.56 ± 1.36, 5.98 ± 1.57, and 6.68 ± 1.58 ng/mL, resp., versus the HFD group, *P* < 0.01, *P* < 0.05, and *P* < 0.01, resp.; Figure 6).

### 3.7. Effects of ECYCD on the mRNA Expression Levels of JNK1, AP-1, IRS-1, and PKB in Liver Tissues

Next, we investigated whether ECYCD affected the mRNA expression of* JNK1*,* IRS-1*,* PKB*, and* AP-1* in the liver. Compared with the control group,* JNK1* and* AP-1* mRNA levels were increased in the HFD group (*P* < 0.01, *P* < 0.01, resp., versus the control group). ECYCD, rosiglitazone, and polyenylphosphatidylcholine inhibited these increases in* JNK1* mRNA expression (*P* < 0.05, *P* < 0.05, and *P* < 0.01, resp., versus the HFD group) and in* AP-1* mRNA expression (*P* < 0.05, *P* < 0.05, and *P* < 0.01, resp., versus the HFD group). Moreover,* IRS-1* mRNA levels decreased in the expression in HFD group (*P* < 0.05, versus the control group), and rosiglitazone significantly increased* IRS-1* mRNA expression (*P* < 0.01, versus the HFD group), whereas ECYCD and polyenylphosphatidylcholine did not affect* IRS-1* mRNA expression (*P* > 0.05).* PKB* mRNA expression in liver tissues did not differ significantly among all groups (*P* > 0.05). These data suggested that the effects of ECYCD on* IRS-1* mRNA and* PKB* mRNA expression were not significant (Figure 7).

### 3.8. Effects of ECYCD on the Levels of JNK1, AP-1, Phospho-IRS-1^ser307^, Phospho-IRS-1^ser307^/IRS-1, Phospho-PKB^ser473^, and Phospho-PKB^ser473^/PKB in Liver Tissues

We aimed to examine whether ECYCD affected the protein expression of JNK1 and AP-1 in the liver by Western blot analysis (Figure 8). Compared with the control group, the HFD group showed increased JNK1 and AP-1 protein expression (*P* < 0.01, for the HFD group versus the control group). JNK1 and AP-1 protein expression levels were significantly reduced in NASH model rats following treatment with ECYCD or polyenylphosphatidylcholine (JNK1: *P* < 0.01, versus the HFD group; AP-1: *P* < 0.05, versus the HFD group). Rosiglitazone significantly inhibited JNK1 protein levels (*P* < 0.05, versus the HFD group); however, no obvious effects were observed on AP-1 (*P* > 0.05, versus the HFD group).

Next, we examined whether ECYCD affected phospho-IRS-1^ser307^, phopsho-IRS-1^ser307^/IRS-1, phospho-PKB^ser473^, and phospho-PKB^ser473^/PKB levels using Western blot analysis. Compared with the control group, phospho-IRS-1^ser307^ levels were significantly increased (*P* < 0.01, versus the control group), and phospho-IRS-1/IRS-1 ratio increased dramatically (*P* < 0.01, versus the control group). ECYCD, rosiglitazone, and polyenylphosphatidylcholine obviously inhibited this increase in phospho-IRS-1^ser307^ levels (*P* < 0.05, versus the control group) and decreased the phospho-IRS-1/IRS-1 ratio (*P* < 0.05, *P* < 0.01, and *P* < 0.05, resp., versus the HFD group). In the HFD group, phospho-PKB^ser473^ levels were markedly decreased when compared with that in the control group (*P* < 0.01, versus the control group). The phospho-PKB^ser473^/PKB ratio was also significantly decreased in the HFD group (*P* < 0.01, versus the control group). ECYCD increased phospho-PKB^ser473^ levels and the phospho-PKB^ser473^/PKB ratio as compared with that in the HFD group (*P* < 0.05, versus the HFD group). Similarly, rosiglitazone elevated phospho-PKB^ser473^ levels (*P* < 0.01, versus the HFD group) and the phospho-PKB^ser473^/PKB ratio (*P* < 0.05, versus the HFD group). However, polyenylphosphatidylcholine did not affect either of these parameters (*P* > 0.05, versus the HFD group; Figure 8).

## 4. Discussion

In the present study, we aimed to determine the curative effects and mechanisms of ECYCD in a rat model of NASH. To this end, we generated a NASH model in rats using a high-fat diet [29, 30]. Increased body weights were observed after 8 weeks of consuming a high-fat diet, and increased body weights, livers weights, and liver indexes were observed after 12 weeks. Histological results indicated that the HFD group showed typical NASH features such as macrovesicular steatosis, ballooned hepatocytes, inflammatory infiltration, and lipid deposition. Consistent with these histological results, serum levels of AST, ALT, TC, TG, and LDL increased dramatically in the HFD group, whereas HDL levels decreased compared with those in the control group. Simultaneously, increases were observed in serum FPG, FINS, and HOMA-IR and liver MDA, FFA, and TNF levels in HFD rats, and decreases were observed in GSH levels. These data indicated that the NASH model was successfully established. Moreover, administration of ECYCD led to decreased body weights, liver weight, and liver indexes. Additionally, dramatic reductions in lipid droplets and inflammatory infiltration were detected in the liver after treatment with ECYCD. Decreases were also observed in AST, ALT, TC, TG, and LDL levels in the serum and in FFAs and TNF in the liver, whereas serum HDL levels increased. These data suggested that ECYCD might affect lipid metabolism and the inflammatory response. FPG and FINS levels and HOMA-IR significantly decreased following the administration of ECYCD, suggesting that ECYCD may alleviate IR. Treatment of ECYCD led to decreased MDA levels in the livers of model rats and increased GSH levels, suggesting that ECYCD may play a role in the antioxidant response. Accordingly, these findings demonstrated that ECYCD had prominent therapeutic effects on rats with NASH.

Next, we further explored the therapeutic mechanisms of ECYCD. Although the etiology of NASH has yet to be fully elucidated, the “two-hit” theory has been accepted as the most popular mechanism [7, 8]. The core element of the “first hit” is IR. IR leads to lipid decomposition and FFA accumulation in the liver. Additionally, lipid degeneration in hepatocytes leads to increased susceptibility of hepatocytes to inflammatory reactions and various injury factors. Previous studies [31] have demonstrated that removing insulin receptor in the muscle or adipose tissue of mice may induce IR, although blood serum glucose levels of mice were normal. After downregulation of the insulin receptor in mouse liver, both blood glucose and insulin levels increased, and IR was observed in the peripheral tissues and liver before systemic IR and hepatic steatosis [13]. These data suggest that the lipid deposition induced by IR in the liver may be the first initiating factor of NASH. IRS is the substrate for the activation of the insulin receptor tyrosine kinase. IRS-1 plays a major role in glucose and lipid metabolism [32, 33]. The insulin receptor is phosphorylated and activates IRS-1 after it binds to insulin. There are some tyrosine phosphorylation sites and serine/threonine phosphorylation sites on IRS-1. When these IRS-1 sites are phosphorylated, the INS signaling pathway is activated, resulting in several biological effects. Abnormal regulation of IRS-1 tyrosine phosphorylation interferes with INS signaling [34, 35], leading to IR. Previous studies have shown that phospho-IRS-1^ser307^ levels and the phospho-IRS-1^ser307^/IRS-1 ratio in the liver were higher than those in healthy control rats [12, 35]. Thus, reducing insulin resistance by reduction of phospho-IRS-1^ser307^ levels and phospho-IRS-1^ser307^/IRS-1 in the liver may be a novel strategy for the treatment of NASH.

Rosiglitazone is an insulin sensitizer and a thiazolidinedione (TZD) drug. Rosiglitazone can improve the sensitivity of target tissues to insulin and reduce IR by activation of PPARs in skeletal muscle, adipose tissue, and liver tissue. As previously reported, rosiglitazone may be an effective treatment for alleviating IR and could reduce lipid deposition in the livers of patients with NASH [36]. Although robust efficacy was demonstrated, further studies are needed to evaluate the drug dose response and long-term safety of this compound. Therefore, it is necessary to identify new methods to reduce IR and lipid deposition in the livers of patients with NASH. In this regard, traditional Chinese medicine has been widely used for the treatment of NASH and has been shown to have curative effects in the treatment of NASH [21]. In our study, we found that ECYCD alleviated IR and lipid deposition in the liver. The protective effects of ECYCD may be attributed to significant regulation of the JNK1 signaling pathway.

JNK1 can be activated by a variety of stimuli, such as the obesity-induced inflammatory response, FFAs, oxidative stress, and endoplasmic reticulum stress (ERS), which may lead to IR and subsequent steatosis in hepatocytes. Previous studies have demonstrated that the JNK1 signaling pathway can be activated in rat livers with high-fat administration for 3 days [37]. However, in a JNK1-knockout rat model, glucose and insulin levels in the serum were decreased significantly [38]. The JNK1 signaling pathway plays a major role in the pathogenesis of NASH. After JNK1 is activated, phospho-IRS-1^ser307^ levels increase through binding of activated JNK1 to IRS-1 and inhibition of IRS-1 tyrosine phosphorylation. Phospho-PKB^ser473^ levels are then decreased further, resulting in attenuation of the INS signal [10–13], eventually leading to IR, hepatic steatosis, and NASH. Hepatic IR can lead to peripheral IR, which results in the decomposition of adipose tissue and increased FFA levels in a vicious feedback cycle [39]. In present study, ECYCD regulated the JNK1 signaling pathway and could reverse the dysregulated expression of key components of the JNK1 signaling pathway, including JNK1, phospho-IRS-1^ser307^, and phospho-PKB^ser473^, thereby inhibiting the activation of the JNK1/phopsho-IRS-1^ser307^/phospho-PKB^ser473^ axis in the JNK1 signaling pathway and alleviating IR and lipid deposition in the liver.

NASH is an important stage in the progression of NAFLD, which is characterized by chronic inflammation of liver tissue and persistent liver damage. The core element of the “second hit” is oxidative stress and lipid peroxidation in the liver. Reactive oxygen species (ROS) are in a state of homeostasis with intracellular antioxidants under normal conditions. Reduced GSH is an important antioxidant in liver cells, and cytochrome P4502E1 (CYP2E1) is the major prooxidant. When NASH occurs, GSH levels in liver cells decrease, and CYP2E1 expression increases, leading to increased levels of intracellular ROS. Through this pathway, JNK1 signaling can be activated, resulting in subsequent activation of the downstream transcription factor AP-1 Y170, release of proinflammatory cytokines, and hepatic inflammation. Inflammatory factors can promote the expression of NADPH oxidase 3 (NOX3) in liver tissue and increase the production of ROS further, thereby aggravating the inflammation and injury of liver tissue. At the same time, ROS can further activate the JNK1 signaling pathway, promoting the release of inflammatory factors [40, 41].

Polyenylphosphatidylcholine has been shown to play a therapeutic role in NASH by regulating the oxidative balance, inhibiting inflammatory factors, alleviating liver injury, and promoting the restoration of liver function [42, 43]. However, similar to rosiglitazone, further studies are needed to elucidate the drug dose response and long-term safety of this drug. In our study, we found that ECYCD also affected the oxidative balance, inhibiting inflammation in the liver and promoting liver function restoration. The protective effects of ECYCD may be attributed to its significant regulation of the JNK1 signaling pathway. Moreover, ECYCD inhibited the activation of the JNK1/AP-1/TNF axis, regulating the oxidative balance, inhibiting inflammation in the liver, and promoting liver function restoration.

In summary, ECYCD had therapeutic effects on rats with high-fat diet-induced NASH through regulation of the JNK1 signaling pathway. ECYCD also alleviated IR and reduced lipid deposition in the liver by blocking the activation of the JNK1/phospho-IRS-1^ser307^/phospho-PKB^ser473^ axis in the JNK1 signaling pathway and regulating the oxidative balance. Furthermore, ECYCD suppressed inflammation in the liver and promoted liver function restoration through the JNK1 signaling pathway. However, our results showed that ECYCD did not affect* IRS-1* mRNA expression, in contrast to previous reports. This may be because of the small sample size used in this study. Accordingly, further studies are needed to compare differences in curative effects and mechanisms between different doses and target agents to test drug target action.

## 5. Conclusions

Our results showed that oral administration of ECYCD could ameliorate high-fat diet-induced NASH in rats. The therapeutic mechanisms may be attributed to significant regulation of the JNK1 signaling pathway. Our study results suggested that ECYCD may be a novel and safe therapeutic option for the treatment of NASH.

## Figures and Tables

**Figure 1:** Effects of ECYCD on body weights (a), liver weights (b), and liver indices (c). Control = control group, HFD = HFD group, ECYCD = ECYCD group, rosiglitazone = rosiglitazone group, and polyenylphosphatidylcholine = polyenylphosphatidylcholine group. Data are presented as the mean ± SD; ^*∗∗*^*P* < 0.01 and ^*∗*^*P* < 0.05 versus the control group; ^#^*P* < 0.05 versus the HFD group (*n* = 10 per group).

**Figure 2:** Histological changes in liver sections in different groups. (a) H&E staining, (b) Oil Red O staining, and (c) the MOD of Oil Red O staining. Arrows in HFD indicate ballooned hepatocytes. Control = control group, HFD = HFD group, ECYCD = ECYCD group, rosiglitazone = rosiglitazone group, and polyenylphosphatidylcholine = polyenylphosphatidylcholine group (*n* = 10 per group). Bar = 400 *μ*m. The MOD of Oil Red O staining in different groups was calculated using Image Pro-plus 6.0 software (MOD = integrated optic density [IOD] sum/area sum). Data are presented as the mean ± SD; ^*∗∗*^*P* < 0.01 versus the control group; ^##^*P* < 0.01 versus the HFD group (*n* = 10 per group).

**Figure 3:** Effects of ECYCD on ALT (a) and AST (b) levels in serum. Data are presented as the mean ± SD; ^*∗∗*^*P* < 0.01 versus the control group; ^##^*P* < 0.01 and ^#^*P* < 0.05 versus the HFD group (*n* = 10 per group).

**Figure 4:** Effects of ECYCD on TG (a), TC (b), HDL (c), and LDL (d) levels in serum. Data are presented as the mean ± SD; ^*∗∗*^*P* < 0.01 versus the control group; ^##^*P* < 0.01 and ^#^*P* < 0.05 versus the HFD group (*n* = 10 per group).

**Figure 5:** Effects of ECYCD on FPG (a) and FINS (b) in serum and on HOMA-IR (c). Data are presented as the mean ± SD; ^*∗∗*^*P* < 0.01 and ^*∗*^*P* < 0.05 versus the control group; ^##^*P* < 0.01 and ^#^*P* < 0.05 versus the HFD group (*n* = 10 per group).

**Figure 6:** Effects of ECYCD on MDA (a), FFAs (b), TNF (c), and GSH (d) in the liver. Data are presented as the mean ± SD; ^*∗∗*^*P* < 0.01 and ^*∗*^*P* < 0.05 versus the control group; ^##^*P* < 0.01 and ^#^*P* < 0.05 versus the HFD group (*n* = 10 per group).

**Figure 7:** Effects of ECYCD on* JNK1* mRNA (a),* AP-1* mRNA (b),* IRS-1* mRNA (c), and* PKB* mRNA (d) expression in the liver. Data are presented as the mean ± SD; ^*∗∗*^*P* < 0.01 and ^*∗*^*P* < 0.05 versus the control group; ^##^*P* < 0.01 and ^#^*P* < 0.05 versus the HFD group (*n* = 10 per group).

**Figure 8:** Effects of ECYCD on JNK1 protein (a), AP-1 protein (b), phospho-IRS-1^ser307^ (c), phospho-IRS-1^ser307^/IRS-1 (d), phospho-PKB^ser473^ (e), and phospho-PKB^ser473^/PKB (f) levels in the liver. Data are presented as the mean ± SD; ^*∗∗*^*P* < 0.01 and ^*∗*^*P* < 0.05 versus the control group; ^##^*P* < 0.01 and ^#^*P* < 0.05 versus the HFD group (*n* = 10 per group).
